# Forecasting COVID-19 Pandemic Using Prophet, ARIMA, and Hybrid Stacked LSTM-GRU Models in India

**DOI:** 10.1155/2022/1556025

**Published:** 2022-05-05

**Authors:** Sweeti Sah, B. Surendiran, R. Dhanalakshmi, Sachi Nandan Mohanty, Fayadh Alenezi, Kemal Polat

**Affiliations:** ^1^Department of Computer Science and Engineering, National Institute of Technology Puducherry, Karaikal, India; ^2^Department of Computer Science and Engineering, Indian Institute of Information Technology Tiruchirappalli, Trichy, India; ^3^Department of Computer Science & Engineering, Vardhaman College Engineering (Autonomous), Hyderabad, Telangana, India; ^4^Department of Electrical Engineering, Jouf University, Sakaka 72388, Saudi Arabia; ^5^Department of Electrical and Electronics Engineering, Bolu Abant Izzet Baysal University, Bolu, Turkey

## Abstract

Due to the proliferation of COVID-19, the world is in a terrible condition and human life is at risk. The SARS-CoV-2 virus had a significant impact on public health, social issues, and financial issues. Thousands of individuals are infected on a regular basis in India, which is one of the populations most seriously impacted by the pandemic. Despite modern medical and technical technology, predicting the spread of the virus has been extremely difficult. Predictive models have been used by health systems such as hospitals, to get insight into the influence of COVID-19 on outbreaks and possible resources, by minimizing the dangers of transmission. As a result, the main focus of this research is on building a COVID-19 predictive analytic technique. In the Indian dataset, Prophet, ARIMA, and stacked LSTM-GRU models were employed to forecast the number of confirmed and active cases. State-of-the-art models such as the recurrent neural network (RNN), gated recurrent unit (GRU), long short-term memory (LSTM), linear regression, polynomial regression, autoregressive integrated moving average (ARIMA), and Prophet were used to compare the outcomes of the prediction. After predictive research, the stacked LSTM-GRU model forecast was found to be more consistent than existing models, with better prediction results. Although the stacked model necessitates a large dataset for training, it aids in creating a higher level of abstraction in the final results and the maximization of the model's memory size. The GRU, on the other hand, assists in vanishing gradient resolution. The study findings reveal that the proposed stacked LSTM and GRU model outperforms all other models in terms of *R* square and RMSE and that the coupled stacked LSTM and GRU model outperforms all other models in terms of *R* square and RMSE. This forecasting aids in determining the future transmission paths of the virus.

## 1. Introduction

Coronavirus is a combination of RNA viruses that usually trigger diseases in animals and birds, but in humans, coronavirus may lead to infections in the respiratory tract. Coronavirus is a Latin word “corona” meaning “crown.” The name coronavirus was given by June Almeida and David Tyrrell in 1930 when they initially noticed and made a study on coronaviruses that infect humans. In 1960, human coronaviruses were discovered [1]. COVID-19 first originated from the region of China, Wuhan, and then transmitted throughout the world. The name COVID-19 was given by WHO (World Health Organization) [2] and was named later SARS-CoV-2 by the International Committee on Taxonomy of Viruses [1]. So far, no particular treatment has been discovered. COVID-19 is a pandemic disease and is generated by the SARS-CoV-2 virus. In 80% of individuals, the pandemic illness is mild, 13% severe, and 6% serious. Fever, fatigue, and a dry cough are the most common symptoms, while others may have body pain, a runny nose, a sore throat, shortness of breath, and diarrhoea [3].

In India, COVID-19 was first detected in Kerala on 20 January 2020 [4]. To raise awareness of the pandemic condition, we proposed a method of forecasting cases using several approaches such as recurrent neural network (RNN), long short-term memory (LSTM), gated recurrent unit (GRU), linear regression, polynomial regression, Prophet, autoregressive integrated moving average (ARIMA), and amalgamated stacked LSTM-GRU. As a result, individuals worldwide may take measures before the number of cases reaches a peak. Awareness can be raised by foreseeing proven cases in advance and holding up a mirror to the real world of a terrible scenario. This awareness can protect the life of a considerable number of people globally if precautions are taken beforehand.

The planned work of the paper is as follows. Analyses of the past study on the COVID-19 dataset using various techniques are given in Section 2.  Section 3 presents the various datasets available on the internet for COVID-19.  Section 4 discusses the methodology.  Section 5 shows the COVID-19 experimental analysis of cases, showing the prediction for the upcoming 20 days using Prophet, ARIMA, and stacked LSTM-GRU.  Section 6 illustrates the challenges faced due to COVID-19 in India overall. Finally, results, conclusion, and future scope are described further in Sections 7 and 8.

## 2. Related Works

The ARIMA model [5] is presented for forecasting confirmed cases. To develop the ARIMA model, a total of 41 days were gathered. In nations such as Italy, China, South Africa, Iran, and Thailand, they utilized the ARIMA model to produce two types of graphs: autocorrelation function graph (ACF) and partial autocorrelation graph (PACF). Finally, a predictive analysis of confirmed instances was displayed. During and after the lockdown period, the corona effect was studied, focusing on positive examples, and the Prophet model, a time series analytic model with superior performance in real-time data, was employed. They discovered that positive instances increased in a regulated manner during the lockdown period compared to the relaxation period, and they argued that the lockdown was justified with strict rules that may prevent the spread of positive cases in India [6]. COVID-19 new and total deaths were analyzed and projected. Time series prediction models such as ARIMA, SARIMA, and Prophet models were used to forecast. The best-fit models were built using the minimum values of Root Mean Square Error (RMSE), Mean Absolute Error (MAE), Akaike Information Criterion (AIC), Mean Square Error (MSE), and Mean Absolute Percentage Error (MAPE). The model's fit was evaluated, and projections for the following 15 to 20 days were created for future usage from these time series models [7–9]. An autoregressive integrated moving average (ARIMA) was used to predict COVID-19 cases based on Johns Hopkins epidemiology data. Between January 20, 2020, and February 10, 2020, the COVID-19 dataset is available. An autoregression (A.R.), a moving average (M.A.), and a seasonal ARIMA model make up the ARIMA model (SARIMA). Differences were favoured to stabilise the time series log transformation. The autocorrelation function (ACF) and partial autocorrelation function (PACF) correlograms were used to test the ARIMA model. ARIMA (1,0,4) outperformed ARIMA (1,0,3) in forecasting COVID-19 incidence, according to the findings.

The incubation duration, count of fundamental regenerations, and a reasonable number of days to cure were all parameters included in the COVID-19 study, which was based on existing Hubei epidemic data. They have also predicted progress in nations like South Korea, Italy, and Iran by presenting existing epidemics and controlling time by tracing transmission dates [10]. Identification of main applications of artificial intelligence for COVID-19 was used to explain COVID-19 analysis. They demonstrate the importance of technology in detecting many instances and forecasting the virus' harmfulness in the next few days by combining and analyzing all primary data. This crucial application was created to keep track of data on recovered, confirmed, or dead patients. The primary role in health monitoring was by A.I. to record the catastrophe of COVID-19 at various scales like epidemiology, medical, and molecular application [11].

COVID-19 has been investigated in nine countries, including India. In COVID-19, they utilized the ARIMA model to forecast the trend. Various ARIMA models were created using various ARIMA parameters, such as ARIMA (3,1,1) models, and the best models were chosen based on the lowest RMSE and MAE values [12]. On the dataset obtained from John Hopkins University repositories, the study of COVID-19 is described using prediction based on two models: SEIR and regression model, with a period of 30th January to 30th March. SEIR and regression models were used to compute and get the real work. Between the regression model and SEIP, the error rate was determined to be 2.01. The illness spread was calculated to be 2.02, which will help the authorities and physicians adjust policy over the next two weeks. These models can tune for predicting long-term intervals using these short-term interval predictions. By retrieving the dataset in a daily layoff, an algorithm can be created in the future to forecast the confirmed case count in a weekly and biweekly period [13].

The topic of the coronavirus' future circumstances was explored. They utilized stacked LSTM, convolutional LSTM, bidirectional LSTM, and month-ahead forecasting. Convolution LSTM outperforms the other two models in terms of forecast accuracy, and the forecast was made with less error [14]. The interplay between various prevalent temperatures in confirmed, suspected, and deceased victims is used to explain COVID-19 analysis. *K*-means clustering was utilized as the machine learning technique, and it was used in the WHO dataset from various parts of China. They discovered that not just the temperature parameter was involved in the circulation of the COVID-19 epidemic after analyzing the information. Future work includes analysis of a whole world dataset of COVID-19 and considering more attributes [15].

Analysis of COVID-19 was explained using an enhanced adaptive neuro-fuzzy inference system (ANFIS) using the Salp Swarm Algorithm (SSA) and Enhanced Flower Pollination Algorithm (FPA). SSA is used in order to avoid the drawback of FPA. The primary purpose of FPASSA-ANFIS was to enhance the performance and is being evaluated using data of WHO (World Health Organization) for future prediction, and also, the model FPASSA-ANFIS was correlated with various other models in order to show good performance as compared to error metrics and computing power [16] and applied six statistical and deep learning algorithms driven by time series techniques to investigate the influence of corona. As a result, ARIMA and TBAT outperformed ARIMA and TBAT in terms of prediction accuracy [17].

COVID-19 analysis is described by predicting released cases, confirmed cases, and death cases on the data using an LSTM-GRU-based RNN model, which produces good results and can undoubtedly recheck the existence of COVID-19 instances. The goal of the recurrent neural network-based model is to provide an automated tool for insisting, assuming the current pandemic scenario, and aiding the government, determining the harshness and health workers to perform for a better decision-making law [18]. The study of COVID-19 was described by utilizing multiple-step prediction to forecast the aggregate confirmed case curves of coronavirus cases across China from 20 January 2020 to 20 April 2020. Combining and subgrouping cities projected the period points of the predicted transmit dynamic curves from January to April 2020 [19].

Shastri et al. [14] evolved an ARIMA model for each nation with a lower RMSE to forecast the evolution of the 145 countries divided into six regions. The ARIMA model allows for the prediction of a virus' behavior. With an RMSE mean value of 144.81, the author postulated a relationship between countries with similar geographic areas and expected COVID-19 cases. As a consequence, the model discovered a correlation between the expected error and the population of each million people. In order to identify the model's optimal parameter, the model was evaluated with 10% of the actual data.

Pandey et al. [13] work is aimed at using LSTM machine learning and GRU in Python to foresee COVID-19 data in Indonesia. Two datasets were utilized as a comparison from other nations with strong associations. The dataset can be found on the ourworldindata.org website. The LSTM model with epoch 15 and an RMSE of 68,417 takes less time to process and is more accurate than the GRU model with an RMSE of 90,173. Indonesian COVID-19 data correlates well with Azerbaijan, Bangladesh, Bhutan, Cape Verde, Curacao, Slovenia, South Africa, and Thailand. The epoch features of LSTM and GRU present a challenge because the amount of COVID-19 data is relatively small.

Bandyopadhyay and Dutta [18] study provided an overview of the major forecasting methods for predicting new COVID-19 cases. In this context, researchers looked at the pandemic's dynamic evolution through time using univariate time series models. Furthermore, incorporating multivariate time series forecasting with weather and daily test data was also used to study the impact of external factors on COVID-19 development. Finally, using MAE, RMSE, and MAPE to analyze the outcomes presented an ensemble learning model based on LSTM and GRU. The results show that the ensemble technique performed well in comparison to other models.

In contrast to these existing approaches, we have proposed a novel hybrid model, which is a stacked LSTM-GRU optimized model. The major goal of the hybrid model is to forecast the COVID-19 cases with improved performance giving better efficiency. This hybrid model is distinct from the existing models in terms of performance and minimum loss while predicting the COVID-19 cases. The model is optimized using Adam optimizer, and the activation function used is ReLu, and the learning rate used is 0.01. Our hybrid model performs better than the Prophet and ARIMA model with minimum loss. Not much work has been done in applying hybrid models to predict COVID-19 cases. It is well known that hybrid models generally perform well over standalone models. So, to enhance the accuracy of the COVID-19 prediction, hybrid models need to be explored.

## 3. Various Dataset Sources of COVID-19

Data is always essential in investigating, studying, and responding to public health emergencies, especially in the situation of a worldwide disaster. Access to datasets and tools to evaluate that data at a large scale is becoming increasingly important in the research process. It is essential in the worldwide response to the new coronavirus. These datasets eliminate obstacles and enable rapid and easy access to vital information, removing the need to search for enormous data files on board. The datasets are available to researchers. These datasets' contents are exclusively made available to the public for educational and research reasons.  Table 1 shows the various other data sources for COVID-19. There are many datasets of COVID-19 available on the internet through various sources as listed below which contain COVID-19 count of cases, text data, radiology pictures, Twitter data, and biological sequences [20].

## 4. Methodology

Kaggle is a great website for learning about machine learning and practicing with R and Python. The best element of Kaggle is the kernel, which assists newbies by bringing everything together in one spot, such as an editor and a dataset with high processing power. Kaggle is the best site for finding datasets on any topic, and it has a variety of COVID-19 datasets. In our proposed work, the dataset is referred from Kaggle (up to 12^th^ Dec 2020), the world's largest dataset repository. This dataset is in .csv format. The dataset has many attributes related to COVID-19 such as date, time, state/union territory, confirmed foreign national, confirmed Indian national, cured, deaths, and confirmed cases. These attributes best describe the COVID-19 cases in India.

Figure 1 represents the per day statistics of cured cases, death cases, and confirmed and new cases in India. The graph is presented up to 12^th^ Dec 2020. The yellow color presents confirmed cases, orange represents death cases, pink represents new cases, and purple represents cured cases. The *x*-axis is labeled as dates, and the *y*-axis is labeled as the number of cases. This graph is represented without the marker value.

Figure 2 mainly focuses on death, cured, and confirmed cases. This graph represents the per day statistics of cases in India with the marker value. The yellow color shows death cases, the green color shows cured patients, and the purple color shows the confirmed cases. The *x*-axis is labeled as to date, and the *y*-axis is labeled as the number of cases.

Figure 3 shows the per day statistics for new cases in India, where the *x*-axis shows the date up to 12^th^ Dec 2020, and the *y*-axis shows the number of new cases. This graph shows the visual view of how daily the new cases are increasing.

### 4.1. Data Analysis Model

The model of data analysis phase includes reading the .csv file, fetching the number of attributes, computing the shape of the dataset, and visualizing the information of the dataset, then grouping the number of confirmed cases, deaths, and cured according to their date and summing them all. Next was retrieving the data of all states and finally plotting the graph for per day statistics in India showing all confirmed, death, and cured cases with marker and without marker values followed by the diagram showing the count of new cases as shown in Figure 4. The visualization and modeling of COVID-19 are crucial and can be extremely useful in the current world condition. Therefore, we used multiple graphs to display the data specifically for India in this paper to assess the trend of COVID-19 growth.

The following are the steps for data analysis:

Step 1: the data analysis phase includes first importing necessary libraries for analyzing the dataset like NumPy, Pandas, matplot, and DateTime.

Step 2: these libraries help the programmer to analyze any data. As the dataset is in .csv format, we import the dataset.

Step 3: we first read the dataset and then store it in pandas data frame.

Step 4: now, the per day statistics graph is plotted to visualize the data. The graph which is used for analysis includes a pie chart and a bar graph.

The infectious disease spreads across communities in predictable ways, which are governed by the pathogen's transmission mechanisms and the relations that the pathogenic agent can employ to propagate around a society. Thus, even small and temporary risks to minute molecules in the air, in confined locations where sufferers breathe, can be acceptable to perpetuate infectious diseases where transmission is forthright from person to person and airborne [23–42].

In Figure 5, the blue color shows confirmed cases, the green color shows the migrated/cured/discharged cases, and the red indicates death cases. Finally, Figure 6 describes the top five states of India that are majorly affected by COVID-19. These bar graphs show the total confirmed cases, cured/discharged/migrated, and death cases.

## 5. Experiment Results and Analysis

Our predictive proposed models are implemented with the required materials as described in Table 2. Table 2 gives the implementation detail of models used.

These models target dividing the population into multiple health states to understand the dynamics of a disease propagation process. The models used are Prophet, ARIMA, and hybrid stacked LSTM-GRU optimized models. The Prophet framework features its data frame, making it simple to work with time series and seasonality data. Two fundamental columns are required in the data frame. “ds” is one of these columns, and it records the date-time series. The relevant values in the time series data frame are stored in the “*y*” column [43].

ARIMA models are statistical models that can be used to examine and forecast time series data. It gives a simple yet powerful way of creating skilled time series forecasts by explicitly catering to a set of common structures in time series data. It is a more complex version of the basic autoregressive moving average that incorporates the concept of integration [44].

The stacked LSTM-GRU optimized hybrid model differs from the existing models in terms of performance and minimum loss while predicting the COVID-19 cases. The model is optimized using Adam optimizer, and the activation function used is ReLu, and the learning rate used is 0.01. Our hybrid model performs better than Prophet and ARIMA models with minimum loss. Not much work has been done in applying hybrid models to predict COVID-19 cases. It is common knowledge that hybrid models outperform standalone models. As a result, hybrid models must be investigated to enhance the performance of the COVID-19 forecast.

### 5.1. Prediction through Prophet

A team on Facebook has released Prophet. This system is used for predicting a series of times. This majorly works well with time series, and it is tough to lose data values and transfer in the trend and outlier [45]. Prophet includes data analysis flow as discussed in Figure 7.

Prophet is an additive regression model. The components of the Prophet model consist of a logistic gain curve trend, and it finds variations in trends by choosing the data's increasing points. A yearly seasonal component can be simulated with the help of the Fourier series. A seasonal weekly element can be represented using dummy variables, and the user can be given a list of holidays [46]. It works well with time series with a lot of seasonal variation and historical data from different seasons. Prophet is forgiving of missing data and trend shifts, and it handles outliers well most of the time [47].

It is given by an equation (Ankit Choudhary et al., 2018):

(1) $$\begin{array}{c} y\left(t\right)=g\left(t\right)+s\left(t\right)+h\left(t\right)+\in_{t}, \end{array}$$

where **g** (**t**) is for demonstrating nonperiodic alterations in period series; the piecewise linear or logistic curve is used. **s** (**t**) are the changes that are done periodically like weekly, yearly, and seasonally. **h** (**t**) is the effect of holidays that the user gives with irregular schedules. ∈_*t*_ is any unusual changes; this is the error term accounts and not accommodated by the model.

Prophet requires the variable names *y* (target) and ds (DateTime) in the time series. Thus, the Prophet model performs best with data from numerous seasons and time series with significant seasonal influences. Furthermore, in comparison to traditional exponential smoothing methods, the Prophet model can extract trends and periodic signals across a wider range of time scales and has no limits on measurement spacing regularity. Thus, the Prophet model simplifies various time series analyses [48].

Some Prophet trend parameters are as follows [49]:

1. *Growth*. Growth is either linear or logistic to show the trend. A piecewise linear curve is fitted over the direction or nonperiodic section of the series to model the trend. The linear fitting procedure shows that spikes and missing data are minimized.
2. *Changepoints*. It includes the list of dates. These changepoints are chosen at random. However, if necessary, a user can manually feed the changepoints. The fit becomes more adjustable as the count of changepoints allowed increases. When working with the trend component, an analyst may encounter one of two issues: overfitting.
3. *Changepoint Prior Scale*. This is the factor for transforming the elasticity of automatic selection on changepoint. A parameter known as the changepoint prior scale could alter the trend flexibility and solve the above two concerns. A higher number will give the time series a more flexible curve.
4. *Daily, Weekly, and Yearly Seasonality*. This contains seasonal patterns like hourly-wise, daily-wise, or yearly-wise data. Prophet uses the Fourier series to fit and forecast the impacts of seasonality and give a flexible model. The Fourier order *N* is an important parameter to choose here, which determines whether more frequency variations can be represented. If the user considers more frequency, components in a time series are just noise.

Figures 8 and 9 show the prediction graph for the number of confirmed and active cases in India from 11^th^ Dec ‘20 to 31^st^ Dec ‘20. The black dots represent the original data values. The blue color line shows the predicted values. The light blue color shows the upper and lower limits for the prediction curve, where ds represent the date and *y* represents the target value of the number of cases in India.

### 5.2. Prediction through ARIMA

This is referred to as the “autoregressive integrated moving average.” It is a model of linear regression. This is also useful for forecasting time sequences. It employs statistical models to forecast future values based on historical data. The notation for this model is as follows: (*p*, *d*, *q*). The autoregression portion of the parameter *p* indicates that it aids in the incorporation of prior ideals into the model means to incorporate the amount of difference in time series, and lastly, *q* is the average running part. This helps in setting the error of the model. This is given by [50, 51]

(2) $$\begin{array}{c} ARIMA\;\left(p,d,q\right)\;\left(P,D,Q\right)\;m, \end{array}$$

where **p** is the order of A.R. term, no. of lags used as a predictor; **d** is the no. of differencing required to make the time series data stationary, if *d* = 0, then stationary; **q** is the order of M.A. term, no. of lagged predicted errors which go into the ARIMA model; **m** is each season of the no. of periods; and (**P**, **D**, **Q**) signifies the periodic section of the time series that is (*p*, *d*, *q*).

ARIMA comprises a data analysis flow as shown in Figure 10, training the data and fitting the ARIMA model by installing the packages. This helps in predicting the next *N* days. Hence, the predicted data can be visualized in a better way.

#### 5.2.1. AR (Autoregression)

The AR, MA, ARMA, and ARIMA models are used to predict the observation at (*t* + 1) using past data from earlier time spots. However, it is vital to ensure that the time series remains stationary over the observation period's historical data. Autoregression (A.R.) is a type of model that calculates the regression of past time series and estimates the current or future values in the series. The moving average (M.A.) model calculates the residuals or errors of past time series and then determines the current or future values in the series. The AR and M.A. models are merged in the ARMA model. For forecasting future data points of the time series, this model considers the impact of previous lags as well as residuals [52].

The mathematical formula for the ARIMA model is given below by [50]

(3) $$\begin{array}{c} y_{t}=\alpha +\beta_{1}\;y_{t}+\beta_{2}\;y_{t-1}+\cdots +\beta_{p}\;y_{t-p}+\epsilon_{1}, \end{array}$$

where *y*_*t*_ are functions of the lags of *y*_*t*_, *α* is the intercept term, *β*_1_ is the coefficient of lag1, and *y*_*t*−1_ is lag1 of the time series.

#### 5.2.2. M.A. (Moving Average)

The mathematical formula is given below by [50]

(4) $$\begin{array}{c} y_{t}=\alpha +\epsilon_{1}+\varphi_{1}\epsilon_{t-1}+\varphi_{2}\epsilon_{t-2}+\cdots +\varphi_{q}\epsilon_{t-q}, \end{array}$$

where *ϵ*_1_ are errors.

In general, the ARIMA model formula can be expressed as [50]

(5) $$\begin{array}{c} \text{Predicted value }y_{t}=\text{constant value}+\text{linear consolidation lags of }Y+\text{linear consolidation of lagged forecast errors}. \end{array}$$

The parameter of the ARIMA model was approximated using the ACF (autocorrelation function) graph and PACF (partial autocorrelation function) [8, 9].

ARIMA shows the prediction of future values in a linear fashion also called the Box-Jenkins model and is given by the equation [53]

(6) $$\begin{array}{c} y_{t}=\theta_{0}+\varphi_{1}y_{t-1}+\cdots +\varphi_{p}y_{t-p}+\in_{t}-\theta_{0}\in_{t-1}-\cdots -\theta_{q}\in_{t-q}, \end{array}$$

where *y*_*t*_ is the actual data point at particular “*t*” time, *θ* and *φ* are the coefficient model, **p** and **q** are form of the autoregressive and moving average, and integer value ∈_*t*_ is an error.

Various steps involved in the ARIMA model are described below [54]:

1. *Checking Stationary*. If the time series has a seasonal component or trend, then before using ARIMA to forecast, it must be made stationary.
2. *Difference*. Through differencing, the time series needs to be stationarized in case of nonstationary. Take as many differences and ensure to check seasonal differences as well.
3. *Filter Out a Validation Pattern*. This is to prove how precise the model is with the use of train test validation.
4. *Select the A.R. and M.A. Terms*. In order to include A.R. term(s), M.A. term(s), or both, use ACF and PACF.
5. *Build the Model*. This includes building the model and setting the duration count to predict *N*, where *N*'s value depends on our needs.
6. *Validate the Model*. This is comparing the forecasted value to the actual value in the validation sample.

Figures 11 and 12 show the prediction graph for the number of confirmed and active cases in India from 11^th^ Dec ‘20 to 31^st^ Dec ‘20. The orange color represents the original data values. The blue color line shows the predicted values, where the *x*-axis represents the date and *y*-axis represents the number of cases in India.

### 5.3. Prediction through Stacked LSTM-GRU Neural Network

LSTM is an exclusive type of RNN introduced by Schmidhuber and Hochreiter [55]. It stands for long short-term memory and is a repetitive network for forecasting the value by learning long observations [56]. LSTM solves the RNN's long-term dependence problem. The input gate, the middle that is the forgotten gate, and the output gate are the three gates of the LSTM. These gates control only the information flow between the cells and the neural structure [57]. The cell state, employed as a carrier of information, is a critical notion in LSTM. Forget gates determine which information should be preserved and which should be discarded. The input gate is used to determine which fresh input, data, and cell state to store. The output gate determines which conditions of the cell become outputs [55].

The stacked model includes data loading, splitting the data into train/test, reshaping data for LSTM, creating the stacked LSTM-GRU model, filling the data into a model, and finally making a prediction, as shown in Figure 13.

The first step is to comprehend the differences between a neural network (N.N.) and a recurrent neural network (RNN), with RNN referring to multilayer neuron networks. Although neural networks are commonly used for classification, grouping, and regression issues, they have one important drawback: they can only use the current input and cannot incorporate the model's prior output. If the input is sequencing input, then we have to consider the previous state also. N.N. do not perform well with sequence input.

Recurrent network handles this problem. It also takes into account the model's current input and prior output. For prediction problems, machine translation, speech recognition, and text summarization, recurrent networks are utilized.

It was initially proposed for language models in 1997. On the output layer of our dataset, a linear regression layer is used (LSTM cell). It is given by [49]

(7) $$\begin{array}{c} h_{1}=H\left(W_{hx}+W_{t}+W_{hx}h_{t-1}+b_{h}\right), \end{array}$$

(8) $$\begin{array}{c} P_{t}=W_{hy}W_{hx}y_{t-1}+b_{y}, \end{array}$$

where **X** = (**x**_1_, **x**_2_, ⋯, **x**_**n**_) denotes the input time series, **h** = (**h**_1_, **h**_2_, ⋯, **h**_**n**_) denotes the hidden state of memory cells, **Y** = (**y**_1_, **y**_2_, ⋯, **y**_**n**_) denotes the output time series, **W** denotes weighted matrices, and **B** denotes the bias vectors.

GRU is an LSTM (long short-term memory) version with only one updated gate consisting of input, forget, and reset gates. Because there is no extra memory cell to store data, it can only control information already within the unit. GRU is a new creation of RNN that is comparable to LSTM in that the update gate is identical to the forget gate and the input gate of LSTM [58]. In this approach, the input and output gates are combined to form a single gate called the update gate. The update gate decides how the unit changes its content by interpolating between prior and candidate activation. Memory modules, rather than hidden units, are used in GRU, ensuring that the gradient does not evaporate or explode after many repeats. The suggested model captures the learning elements of both the LSTM and GRU models due to its ability to capture the distinct benefits of both models in a single framework. The GRU model, which processes the time series data, uses the stacked LSTM output as an input. The GRU model's generated output represents the output of the hybrid stacked LSTM and GRU model. Using stacked LSTM in a neural network to improve prediction accuracy while learning a large number of temporal features is a frequent practice. They also help to generate a better level of representation of the incoming sequence data over time. Although the stacked model requires a large dataset for training, it aids in increasing the model's memory size [59].

Now, the curve in Figure 14 shows the train prediction and test prediction (8 : 2) with the original curve.

Figures 14 and 15 show the prediction graph for the number of confirmed and active cases in India from 11^th^ Dec ‘20 to 31^st^ Dec ‘20. The blue color represents the original data values. The orange color line shows the trained values. The green color shows the prediction curve, where the *x*-axis represents the date and *y* represents the number of cases in India. The dataset was divided into train and train ratio that is 8 : 2. Further, the hybrid model is optimized using Adam optimizer for more accurate results.

### 5.4. Adam Optimizer and Activation Function

With the inclusion of momentum, Adam is a cross between RMSprop and stochastic gradient descent. It uses squared gradients to scale the learning rate, similar to RMSprop. However, it uses a moving average of the gradient rather than the gradient itself to take advantage of momentum, identical to SGD with momentum. Adam is a learning rate algorithm that calculates individual learning rates based on a variety of variables. Adam uses adaptive moment estimation to modify the learning rate for each weight of the neural network by estimating the first and second moments of the gradient [60]. When constructing your neural network, the learning rate may be the most crucial hyperparameter. As a result, it is critical to understand how to examine the effects of the learning rate on model performance and to develop an intuition for the learning rate's dynamics on model behavior [8, 61]. Because the derivative of the ReLu function is 1 for positive input, it can help deep neural networks train faster than typical activation functions. As a result, deep neural networks do not require additional time during the training phase to compute error terms due to a constant [62].

### 5.5. Comparison between Prophet, ARIMA, and LSTM-GRU

The comparison between models are specified below [43, 47, 48, 50, 51, 59, 63]:

1. ARIMA is a type of autoregressive forecasting in which the lag values and error terms are used to fit a linear regression line. Facebook's FbProphet is known for being simple to use but challenging to master, especially if you want to learn more about what is going on with the model. The Fourier transform is at the heart of it
2. Before utilizing ARIMA, you must have a basic understanding of statistics. You can achieve a reasonable forecast on messy data using FbProphet with no manual effort
3. ARIMA is susceptible to white noise and nonstationary signals, whereas FbProphet is resistant to outliers, missing data, and significant changes in your time series
4. The autoregressive component *p*, the integrated component *d*, and the moving average component *q* can all be experimented with in ARIMA. Linear or logistic growth, holidays, seasonalities, and changepoints are all parameters that can be experimented with in FbProphet
5. The autocorrelation function (ACF) and partial autocorrelation function (PACF) graphs can be used to find correct values for *p* and *q* while tuning an ARIMA model. Tuning the “*n* changepoints” parameter in FbProphet helps the model catch the trend in the training data. The large number of “*n* changepoints” may result in model overfitting, lowering the model's prediction accuracy on new data
6. The GRU model, which processes the time series data, uses the stacked LSTM output as an input. The GRU model's generated output shows the output of the hybrid stacked LSTM and GRU model. Using stacked LSTM in a neural network to improve prediction accuracy while learning a large number of temporal features is a frequent practice. They also help to generate a better level of representation of the incoming sequence data over time

## 6. Challenges Faced due to COVID-19 in India

There are several challenges faced due to the impact of COVID-19 in overall India. Few are given below [64]:

1. The COVID-19 pandemic has wreaked havoc on the construction industry, which is particularly vulnerable to economic cycles
2. The COVID-19 pandemic has raised attention to the already overburdened and understaffed home and institutional-based care systems in various nations. This short highlights the issues of recruiting, deploying, retaining, and protecting a sufficient number of well-trained and motivated care workers
3. The COVID-19 epidemic is wreaking havoc on public health and wreaking havoc on the economy and labor market, particularly for forest workers and enterprises. It has exacerbated existing issues, and as a result, many businesses and workers have suffered
4. As individuals can freely move across jurisdictions and countries, the road transportation business is vital to social and economic development. In an attempt to curb the spread of COVID-19, numerous nations worldwide have implemented domestic transit restrictions and/or closed border crossings for road freight transportation services. However, if the crisis is to be adequately handled, governments, social partners, and parties involved in the road transport supply chain—such as shippers, receivers, transport purchasers, and middlemen—must act rapidly to solve the issue of decent work for these critical individuals
5. Due to a combination of aircraft cancellations and restrictions aimed at preventing the spread of COVID-19, international travel has practically ground to a halt
6. Tourism is a significant source of job creation and economic development. COVID-19, on the other hand, has made a considerable difference. The impact on tourism businesses and workers, the majority of whom are young women, is unprecedented
7. As the disease develops, food delivery networks must remain operational to avoid a food crisis and reduce the worldwide economic impact
8. Even though many teachers in developing countries lack the essential skills and equipment to conduct successful remote education, most instructors and their organizations have accepted this challenge

## 7. Results and Conclusion

As a result, we investigated various forecasting models critical to illness prediction and demonstrated the expansion of COVID-19 cases in India. The prediction values from the hybrid model are more fit than the state-of-art models, as evidenced by the above data and line plots. These forecasted numbers are for the next few days. When the predictive values rise, the number of new cases will increase as well. Humans would have to battle the coronavirus in the future and obey the Government of India's guidelines. Our models are capable of forecasting instances for the following 20 days and even farther ahead, as shown in Table 3. Table 3 shows the statistical values for forecasted COVID-19 new confirmed cases in India.

Finally, the graphs of these models were compared, and the findings revealed that the stacked LSTM-GRU prediction was superior to the state-of-the-art models, as shown in Table 4. Hence, the characteristics of good predicting models should fit the past data value and be simple but effective. The state-of-the-art model taken is linear regression, polynomial regression, LSTM, GRU, RNN, ARIMA, and Prophet. Table 4 shows the performance metrics for various models showing comparison with the state-of-the-art models.  Table 5 indicates the evaluation metrics.

As a result, as shown in Table 4, we investigated several models such as the recurrent neural network (RNN), gated recurrent unit (GRU), long short-term memory (LSTM), linear regression, polynomial regression, autoregressive integrated moving average (ARIMA), prophet, and hybrid stacking LSTM-GRU. The Root Mean Square Error (RMSE) is a quadratic scoring technique for calculating the mean magnitude of an error. To put it another way, the difference between the predicted and actual values is squared before being averaged over the sample value. Finally, the square root value of the average is determined. A lower RMSE value indicates that the model performs better [66]. It indicates how effectively the regression line predicts real-world values by the degree to which a data point fits the linear regression. You may calculate the amount of variance presented by the model's self-standing variables using the coefficient of determination. It determines the model's goodness-of-fit and assigns a score between 0 and 1 to it [67].

## 8. Future Works

The majority of current instances in India are asymptomatic, indicating that the person is infected but does not show any symptoms of coronavirus infection. The disease's name is COVID-19, and it is a terrible one. The virus must be well understood by the public. In proportion to our population, India's new occurrence figures are not as alarming at the time. This is only possible through a series of lockdowns. The information gathered in this study was compared to confirmed daily COVID-19 cases in India. According to the data, the daily number of cases in India is likely to approach 1,500,000 instances per day in the next four weeks. Based on the dataset, this prediction was created in light of the current circumstances. While forecasting is not flawless, it can undoubtedly be used as a preventative measure. Future work can be improved by combining new components and algorithms with the hybrid model to generate more accurate findings.

## Figures and Tables

**Figure 1:** Per day statistics of India (considering all cured cases, death cases, confirmed cases, and new cases), where the *x*-axis is “date” and *y*-axis represents “number of cases.”

**Figure 2:** Per day statistics of India with marker values showing no. of confirmed, cured, and death cases.

**Figure 3:** Per day statistics for new cases in India.

**Figure 4:** Model of the data analysis phase.

**Figure 5:** Bar graph showing the percentage of confirmed/cured/death cases per state (India).

**Figure 6:** Top five states of India (cases of COVID-19).

**Figure 7:** Working model of Prophet.

**Figure 8:** Prediction through Prophet for a count of confirmed cases (for the next 20 days), where the *x*-axis is “ds” and *y*-axis is “*y*” which is the target.

**Figure 9:** Prediction through Prophet for the number of new cases (for the next 20 days), where *x*-axis is “ds” and *y*-axis is “*y*” which is target.

**Figure 10:** Working model of ARIMA.

**Figure 11:** Prediction through ARIMA for the confirmed cases (for the next 20 days), where the *x*-axis is “dates” and the *y*-axis is “total cases.”

**Figure 12:** Prediction through ARIMA for the new cases (for the next 20 days), where the *x*-axis is “dates” and the *y*-axis is “total cases.”

**Figure 13:** Model of stacked LSTM-GRU.

**Figure 14:** Prediction through stacked LSTM-GRU neural network for new cases (for the next 20 days), where the *x*-axis is “days” and the *y*-axis is “number of cases.”

**Figure 15:** Prediction curve for confirmed cases, where the *x*-axis shows “days” and *y*-axis shows the “number of cases.”

**Table 1:** Various other data sources for COVID-19.

Data source	Type of data	Link
WHO	This dataset is provided by WHO (World Health Organization), providingup-to-date data across the world. This is the official website to get the COVID-19 case live updates and get information about outbreaks	https://systems.jhu.edu/research/public-health/ncov/
Kaggle	Kaggle is the largest data science community to provide an open-source dataset globally. Every day, the count of new cases increases around the world. This collection contains data from India's states and also union territories on a daily basis	https://www.kaggle.com/sudalairajkumar/covid19-in-India
Johns Hopkins University	Johns Hopkins University's Center for Systems Science and Engineering team maintains the dashboard and dataset (CSSE). Since January 22, 2020, it has been posting data on confirmed cases and deaths for all nations. Every day, JHU updates its data many times. This information comes from governments and national and subnational agencies all across the world; a complete list of data sources for each country may be seen on the Johns Hopkins GitHub page. It also makes its data available to the general public there [21]. This provides public access for testing data, resources, and analysis. Web-based outline for cases globally	https://systems.jhu.edu/research/public-health/ncov/
C. R. Well's GitHub	Open-source, writable linked data repository, developed by Thomson Reuters and Refinitiv and is used as a central knowledge graph database [22]	https://github.Com/WellsRC/Coronavirus-2019
China CDC (CCDC)	This dataset shows the daily count of cases particularly in China consisting of confirmed, asymptomatic, and recoveries	http://weekly.chinacdc.cn/news/Trackingtheepidemic.htm
DataHub	DataHub provides time series data on COVID-19 cases. The data is in .csv format and is updated on a daily basis. It comes from this upstream repository, which is managed by the fantastic team at Johns Hopkins University's Center for Systems Science and Engineering (CSSE), who have been collecting data from all around the world since the beginning	https://datahub.io/core/covid-19
Conference of State Bank Supervisors	This provides a country-level map of COVID cases in the U.S., which is revised hourly	https://www.csbs.org/information-covid-19-coronavirus
U.S. CDC	This provides the cases in U.S. Consumers, financial institutions, and fellow regulators will get timely information on actions taken to support communities during the COVID-19 epidemic from state regulators. This website will be updated with all public CSBS updates related to COVID-19	https://www.csbs.org/information-covid-19-coronavirus
Italy Ministry of Health	This provides the COVID-19 cases in Italy	https://www.salute.gov.it/portale/nuovocoronavirus/homeNuovoCoronavirus.jsp
U.S. National Institutes of Health	This provides overall COVID-19 cases in the U.S.	https://covid19.nih.gov/
W. Zeng's website	This website provides the global COVID-19 cases country-wise	http://open-source-covid-19.weileizeng.com/
COVID-19 Radiography Database	This provides COVID-19, 45k scholarly articles, and its family. This publicly available dataset is made available to the world's researchers to use recent developments in natural language processing (NLP) and other A.I. approaches to bring about fresh intuition in support of the ongoing fight against this disease	https://www.kaggle.com/allen-institute-for-ai/CORD-19-research-challenge
A. G. Chung's GitHub—Actualmed Initiative	It includes an X-ray image dataset of the chest initiative of COVID-19	https://github.com/agchung/Figure1-COVID-chestxray-dataset/tree/master/images
Georgia State University's Panacea Lab	This chatter in Twitter provides the different linguistic datasets. The data obtained from the stream includes all languages, but English, Spanish, and French have the highest incidence	http://www.panacealab.org/covid19/
NCBI GeneBank	This provides the sequence of SARS-CoV-2	https://www.ncbi.nlm.nih.gov/sars-cov-2/
The GISAID Initiative	This is the global proposal revealing all types of cold data	https://www.gisaid.org/
China National GeneBank	This provides the sequence database of COVID-19	https://db.cngb.org/datamart/disease/DATAdis19/
EMBL-EBI	This provides the sequence of COVID outbreak isolates and record	https://www.covid19dataportal.org/

**Table 2:** Implementation detail of models used.

Dataset used	COVID-19 Indian dataset from Kaggle (up to 12^th^ Dec 2020)
Models used	Prophet, ARIMA, stacked LSTM-GRU
Language	Python
System software	Co-Lab
Libraries used	Pandas, NumPy, Sklearn, Matplotlib, FbProphet, ARIMA, LSTM, Sequential, Dense, Math, DateTime

**Table 3:** Statistical values for forecasted COVID-19 new confirmed cases in India.

Date	Forecasted COVID-19 new confirmed cases
11/12/2020	29,340
12/12/2020	26,819
13/12/2020	31,100
14/12/2020	27,546
15/12/2020	22,051
16/12/2020	26,111
17/12/2020	24,000
18/12/2020	22,700
19/12/2020	21,354
20/12/2020	29,456
21/12/2020	34,567
22/12/2020	23,965
23/12/2020	24,700
24/12/2020	23,765
25/12/2020	24,567
26/12/2020	27,912
27/12/2020	18,722
28/12/2020	16,400
29/12/2020	19,500
30/12/2020	21,800
31/12/2020	21,121

**Table 4:** Performance metrics for various models showing comparison with the state-of-the-art models.

Performance metrics	RNN	GRU	LSTM	Linear regression	Polynomial regression	ARIMA	Prophet	LSTM-GRU
*R* square	0.30	0.74	0.05	0.01	0.31	0.56	0.46	0.74
RMSE	120.35	94.558	134.505	284809.4	149117.8	1260	568.58	69.92

**Table 5:** Evaluation metrics.

*R* ^2^	$R^{2}=1-\left(\frac{\sum {\left(Y_{i}-X_{i}\right)}^{2}}{\sum {\left(Y_{i}-Z_{i}\right)}^{2}}\right)$	Where *Y*_*i*_ is the actual value at certain *i*^th^ assumption, *X*_*i*_ is the forecasted value at *i*^th^ assumption, *Z*_*i*_ shows the average of the overall observations, and *n* is the total count of observations
RMSE	$\text{RMSE}=\sqrt{\sum \frac{{\left(Y_{i}-X_{i}\right)}^{2}}{n}}$	Where *Y*_*i*_ shows the forecasted value, *X*_*i*_ shows the true value, and *n* is the count of observations [65]

## Data Availability

We can send the datasets at the request of the authors.
